This article has been retracted.

# Hypoxia Tumor Microenvironment Activates GLI2 through HIF-1*α* and TGF-*β*2 to Promote Chemotherapy Resistance of Colorectal Cancer

**DOI:** 10.1155/2022/2032895

**Published:** 2022-02-10

**Authors:** Kun Huang, Xin Zhang, Yanhui Hao, Ruixing Feng, Haojie Wang, Zhiwan Shu, An Li, Minghu Du

**Affiliations:** ^1^Department of General Surgery, Central Hospital of Jiangjin District, Chongqing, China; ^2^Research Center of Basic Medical Science, Medical College of Qinghai University, China; ^3^Department of Radiation Oncology, Affiliated Hospital of Qinghai University, China; ^4^Affiliated Hospital of Qinghai University, China; ^5^Department of Neurology, Zhengzhou Central Hospital, Xinxiang Medical College, China; ^6^Wuwei City People's Hospital, China

## Abstract

**Background:**

A majority of relapse cases have been reported in colorectal cancer patients due to cancer stem cell progenitors. The factors responsible for chemoresistance have yet to be discovered and investigated as CSCs have reported escaping from chemotherapy's killing action.

**Objective:**

In this study, we have investigated the effects of HIF-1*α* and TGF-*β*2 in hypoxia conditions on the expression of GLI2, which is a potential factor for causing chemoresistance. *Material and Methods*. Colorectal samples of treated patients were collected from the Hospital Biological Sample Library. Culture of patient-derived TSs and fibroblasts was performed. The collected patient samples and cells were used for immunohistochemistry, quantitative PCR, and western blotting studies which were performed.

**Results:**

It was reported that HIF-1*α* (hypoxia-inducible factor) and TGF-*β*2 secreted from cancer-associated fibroblasts (CAFs) synergistically work to express GLI2 in cancer stem cells. Hence, it increased the stemness as well as resistance to chemotherapy.

**Conclusion:**

The HIF-1*α*/TGF-*β*2-mediated GLI2 signaling was responsible for causing chemoresistance in the hypoxia environment. High expressions of HIF1*α*/TGF-*β*2/GLI2 cause the relapsing of colorectal cancer, thus making this a potential biomarker for identifying the relapse and resistance in patients. The study uncovers the mechanism involved in sternness and chemotherapy resistance which will help in targeted treatment.

## 1. Introduction

Colorectal cancer is a significant cause of cancer deaths worldwide due to the prominent resistance mechanisms which further add to the disease progressions [1]. The resistance is caused due to clone drug targets which upregulate many pathways.

Colorectal cancer is also diagnosed worldwide, affecting around 1.4 million people, of which approximately 700,000 patients have reportedly died [2]. Surgery, chemotherapy, and radiotherapy are amongst the most opted methods for treating colorectal cancer. Due to the high prevalence, fast progression, and recurrence of this disease [3, 4], current demands are focused on developing new treatment options for better efficacy. Currently, cisplatin is a popular choice of drugs amongst physicians for first-line therapy [5].

But in the current scenarios, many cases of chemoresistance have been noted in the cisplatin therapies due to many other factors yet to be discussed [6]. Intratumoral hypoxia regions devoid of oxygen supply are a prominent factor in developing paced growth in solid tumors [7].

HIF-1*α* (hypoxia-inducible factor 1 alpha) has been reported to promote tumors in many conditions [8]. In breast cancer, HIF-1*α* was able to activate MMP9 (matrix metallopeptidase 9). HIF-1*α* is also regulated by binding with hypoxia response element (HRE) [9]. In hepatocellular carcinoma studies, HIF-1*α* was found to activate SNAIL1.

Amongst the stromal factors, colorectal cancer cell-derived TGF-*β* has shown the stimulation of cancer-associated fibroblasts (CAFs), thereby causing secretion of interleukins (IL-11), which leads to triggering of the GP130/STAT3 signaling in CRCs. Thus, programs involving TGF-*β*-induced stromal gene expression are good predictors of metastasis and recurrence in colorectal cancer cells (CRCs) [10, 11].

## 2. Material and Methods

### 2.1. Culture of Patient-Derived TSs and Fibroblasts

Samples of treated patients were collected from the Hospital Biological Sample Library after receiving ethical approval for research from the committee at the hospital in China. Institutional Research Board approved all the studies. Human colon samples collected from the hospital library were minced and thoroughly digested using 1 mg mL^−1^ of collagenase (Thermo Fisher) at 37°C in Dulbecco's modified Eagle medium/Nutrient Mixture F-12 (DMEM/F-12) for 1 hour. Then, the cells were cultured using a CSC medium. TSA cells were generated and then resuspended.

In fibroblast isolation, colorectal samples and mucosal cells were minced and incubated for thirty minutes at 37°C. The epithelial cells were removed by rigorous shaking. Fibroblasts were harvested after collagen removal by collagenase.

### 2.2. Histological and Immunohistochemical Analysis

Samples were collected from rats fixed with 4% paraformaldehyde in phosphate-buffered saline overnight. They were then embedded in paraffin wax. 5 *μ*m sections were cut off and stained using hematoxylin and eosin.

The expressions of HIF-1*α* were checked using IHC analysis. Positive staining of more than 10% of cancer cells was considered positive. Staining positively stained cells against the total tumor cells was used for quantitative analysis. To reduce the observational bias, two pathologists verified the positive cell counting.

### 2.3. Western Blot Analyses

1% NP-40 lysis buffer was used to lyse cells from 10 cm dishes for thirty minutes on ice. SDS-PAGE was used to separate proteins and then transferred to the nitrocellulose membrane. These membranes were incubated with primary then secondary antibodies. *β*-Actin was used for internal control.

### 2.4. RNA Preparation and Real-Time PCR

TRIzol Reagent (Thermo Fisher) was used to extract RNA, and PrimeScript™ (Cytiva Life Sciences) was used to isolate 1 *μ*g cDNA as per the manufacturer's instructions. qRT-PCR was performed using ABI PRISM 7000 (Thermo Fisher) via Direct RT-qPCR Kit (Cytiva Life Sciences).

### 2.5. Tissue Specimens

Human colorectal cancer tissue microarrays, as well as CRC tissue samples, were collected from the Hospital Biological Sample Library. The review board approved the studies. Informed consent was approved for those patients who agreed to participate in the study.

### 2.6. Statistical Analysis

GraphPad Prism 6 software was used for performing statistical analysis. The values were expressed as the mean ± SD. Analysis was performed where *P* value < 0.05 was considered as significant.

## 3. Results

### 3.1. Cancer-Associated Fibroblasts and Hypoxia Promote Chemotherapy Resistance via GLI2

The role of cancer-associated fibroblasts (CAFs) and tumorsphere (T.S.) interactions was studied in hypoxia conditions which promoted chemoresistance. The tumorsphere was infected with luciferase for analyzing its viability for T.S. cells. It was noted that the tumorsphere (T.S.), when compared with TS-derived adherent cells (TSA), was lesser in the 5-Fu and oxaliplatin (FOLFOX) regimen. The treatment of tumorsphere cells with CAF-CM and TGF-*β*2 led to resistance which was not seen in IL-6, Wnt3a, and Wnt5a treatments (Figure 1).

When cocultured, TS-derived adherent cells (TSA) and tumorshpere (T.S.) showed an increase in chemotherapy (Figure 2).

Hypoxia was reportedly increasing the resistance in tumorsphere cells against chemotherapy when cocultured with cancer-associated fibroblasts (CAFs). HIF-1*α*, TGF-*β*2, and GLI2 expressions define the outcomes in colorectal cancer. The immune histochemistry was studied for cells for quantification of expressions of GL12 and its correlation with HIF-1*α* and TGF-*β*2 (Figure 3).

### 3.2. Immunofluorescence

Immunofluorescent assay shows the fluorescence of GLI proteins or nucleus (DAPI) in TS1-CAFs coculture stained with DAPI, caspase, and BrDU for both normoxia and hypoxia environments at 24 hours.

### 3.3. Reversing Chemoresistance

The combinational therapy of GANT61 (GLI inhibitor) and SD208 (TGF-*β* inhibitor) has effectively reversed the chemoresistance. The pathway used for reversing the chemoresistance was the TGF-*β*/GLI2 pathway, where GANT61 and SD208 blocked the DNA binding activity of transcription factors GLI1/2. The tumorsphere cells were grown in a cancer-associated fibroblast conditional medium (Figure 4).

This also suggests that the TGF-*β* signaling via GLI2 modulates the apoptosis and survival of cells, affecting the cell differentiation process. The experimentation also noted that TGF-*β* in hypoxia treatment affected the PARP and caspase 3 activation, which was the opposite of GANT61, supporting the role of TGF-*β*/GLI2 in the modulation of apoptosis.

Hence, it was confirmed that the combinational treatment of SD208 and GANT61 targeted TGF-*β*-mediated differentiation and survival, causing synergistic effects for inducing chemoresistance. The combinational therapy of SD208 and GANT61 with inhibitors caused the resensitization of TS1 and TS2 cells in the hypoxia environment of CAF. This therapy was effective in comparison to SD208 or GDC0449 alone.

### 3.4. Hypoxia Environment in Cancer-Associated Fibroblasts Induces GLI Expressions with the Combinational Effect of HIF-1*α* and TGF-*β*2

Hypoxia that leads to chemoresistance is a well-resonated hypothesis; the role of TGF-*β*2-GLI2 activity in CAF-mediated cells and tumor reoccurrence was further investigated. Immunostaining was done to assess the expressions of GLI2 proteins in the tumorsphere cells, which were being cocultured with cancer-associated fibroblasts (CAFs) (Figure 5). Even the tumorsphere cells, when exposed to a hypoxia environment, have shown an increase in mRNA expression of GLI2 protein, which was further confirmed with elevation on receiving TGF-*β* treatment (Figures 6 and 7). Western blotting was also performed which induced GLI2, hence confirming the analysis of TGF-*β* treatment under a hypoxia environment (Figure 8).

Mean intensity of GLI2 fluorescence and IHC has shown the coordination of TGF-*β* with hypoxia for inducing GLI2.

## 4. Discussion

The mechanism of chemoresistance in the environment of hypoxia has shown that this condition of hypoxia regulates the colorectal cancer cell plasticity, thereby helping them escape the killing action of chemotherapy. The study mainly focused on understanding patient models and the relevance of hypoxia and its correlation with cancer-associated fibroblasts (CAFs) and cancer stem cells.

Cancer-associated fibroblasts are the major tumor microenvironment factors responsible for generating and releasing potential factors for tumor malignancy [12]. Many studies have been performed for understanding the signaling mechanisms that cause chemoresistance. In the studies conducted, it was found that cancer-associated fibroblast activation caused secretion of interleukin-11, which caused further activation of CRC. The results from the hypoxia conditions have shown that the tumor environment has significantly caused chemoresistance. It was also found that synergistically, the expressions of GLI2 were induced by HIF-1*α* and TGF-*β* signaling. Both were responsible for inducing chemoresistance. Cancer-associated fibroblasts have also been reported to increase TGF-*β* cytokine levels, promoting cancer stem cells (CSC) even in a chemotherapy environment. This further strengthens the role of the TGF-*β* signaling under hypoxia conditions for promoting expressions of GLI2 and chemoresistance.

## 5. Conclusion

This study concluded that the expressions of GLI2 were increased due to CAF-secreted TGF-*β* which promoted the stemness in colorectal cancer cells, thus causing chemoresistance. It was also found that no signs of Wnt signaling as a crucial factor were needed to mediate CAF-enhanced CSC. Wnt3a or Wnt5a failed to generate any induction of the colorectal stem cell genes while TGF-*β* induced it strongly.

### 5.1. Further Studies

It was speculated that further studies must be done to study the intrinsic action of Wnt signaling pathways for self-renewal action, which might be a factor to explore in this microenvironment. New studies must elaborate the role of inhibitors of TGF-*β* to control chemoresistance in humans.

## Figures and Tables

**Figure 1:** Cancer-associated fibroblasts (CAFs) in hypoxic environment induce chemoresistance in a GLI2-dependent manner. The cell viability was checked where the cells were both left treated and untreated with CAF conditional medium which was followed by administration with chemotherapeutic reagents for other five days.

**Figure 2:** The cell viability of T.S. with or without cancer-associated fibroblasts (CAFs) for 72 hours with combinational therapy of chemotherapeutic agents for again 72 hours.

**Figure 3:** Immunohistochemical staining done and normal versus hypoxia conditions were studied where tumorsphere cells from patients without any cancer-associated fibroblasts (CAFs) showed only modest effects. Hence, this further confirms that the CAFs in hypoxia coordinate synergistically to increase level of chemotherapy resistance.

**Figure 4:** Quant. PCR analysis showing expressions of cancer stem cells and stemness genes in combination treatment with SD208 and GNT61. It reversed the chemoresistance in the tumor microenvironment.

**Figure 5:** Immunofluorescence analysis of GLI proteins and DAPI nucleus under both normal and hypoxia conditions for quantification and analysis of proteins in 24 hours.

**Figure 6:** GLI2 expressions were quantified in both TS1A and TS2A with or without TGF-*β*2 in normal or hypoxia for 48 hours.

**Figure 7:** Mean GLI2 fluorescence protein intensity.

**Figure 8:** Cell viability was assessed with/without cancer-associated fibroblasts for 7 days in both normoxia or hypoxia environments when combined with chemotherapy treatments for seven days. In the western blot, cell viabilities of tumorsphere with three shGLI2-A, B, C were checked independently.

## Data Availability

The data could be obtained by contacting the corresponding author.

## References

[1] Dienstmann R., Vermeulen L., Guinney J., Kopetz S., Tejpar S., Tabernero J. (2017). Consensus molecular subtypes and the evolution of precision medicine in colorectal cancer. *Nature reviews cancer*.

[2] Peng H., Wang L., Su Q., Yi K., du J., Wang Z. (2019). miR-31-5p promotes the cell growth, migration and invasion of colorectal cancer cells by targeting NUMB. *Biomedicine & Pharmacotherapy*.

[3] Suehiro Y., Takemoto Y., Nishimoto A. (2018). Dclk1 inhibition cancels 5-FU-induced cell-cycle arrest and decreases cell survival in colorectal cancer. *Anticancer Research*.

[4] Nakurte I., Jekabsons K., Rembergs R. (2018). Colorectal cancer cell line SW480 and SW620 released extravascular vesicles: focus on hypoxia-induced surface proteome changes. *Anticancer Research*.

[5] Zhang L., He L., Zhang H., Chen Y. (2018). Knockdown of miR-20a enhances sensitivity of colorectal cancer cells to cisplatin by increasing ASK1 expression. *Cellular Physiology and Biochemistry*.

[6] Xie T., Li Y., Li S. L., Luo H. F. (2016). Astragaloside IV enhances cisplatin chemosensitivity in human colorectal cancer via regulating NOTCH3. *Oncology Research*.

[7] Semenza G. L. (2010). HIF-1: upstream and downstream of cancer metabolism. *Current Opinion in Genetics & Development*.

[8] Higgins D. F., Kimura K., Bernhardt W. M. (2007). Hypoxia promotes fibrogenesis in vivo via HIF-1 stimulation of epithelial-to-mesenchymal transition. *The Journal of Clinical Investigation*.

[9] Choi J. Y., Jang Y. S., Min S. Y., Song J. Y. (2011). Overexpression of MMP-9 and HIF-1*α* in breast cancer cells under hypoxic conditions. *Journal of Breast Cancer*.

[10] Sadanandam A., Lyssiotis C. A., Homicsko K. (2013). A colorectal cancer classification system that associates cellular phenotype and responses to therapy. *Nature Medicine*.

[11] de Sousa E Melo F., Wang X., Jansen M. (2013). Poor-prognosis colon cancer is defined by a molecularly distinct subtype and develops from serrated precursor lesions. *Nature Medicine*.

[12] Su S., Chen J., Yao H. (2018). CD10^+^GPR77^+^ cancer-associated fibroblasts promote cancer formation and chemoresistance by sustaining cancer stemness. *Cell*.

